The article "Preventive Electroacupuncture Alleviates Oxidative Stress and Inflammation via Keap1/Nrf2/HO-1 Pathway in Rats with Cyclophosphamide-Induced Premature Ovarian Insufficiency" was retracted in 2023. Reasons: unreliable results or conclusions; concerns about the data; concerns about the peer review; concerns about the citations.

# Preventive Electroacupuncture Alleviates Oxidative Stress and Inflammation via Keap1/Nrf2/HO-1 Pathway in Rats with Cyclophosphamide-Induced Premature Ovarian Insufficiency

**DOI:** 10.1155/2022/6718592

**Published:** 2022-08-25

**Authors:** Yang Chen, Rui Zhao, Xiang Li, Yun-peng Luan, Li-wei Xing, Xiao-juan Zhang, Jing Wang, Xiao-yan Xia, Rong Zhao

**Affiliations:** ^1^Nanjing University of Chinese Medicine, Nanjing 210023, China; ^2^Department of TCM, Hainan Women and Children's Medical Center (Women and Children's Health Care Center of Hainan Province, Hainan Children's Hospital, Children's Hospital of Fudan University at Hainan, Hainan Obstetrics and Gynecology Hospital), Longkun Road, Qiongshan District, Haikou, 571100 Hainan, China; ^3^Yunnan University of Chinese Medicine, Kunming, 650500 Yunnan, China; ^4^Southwest Forestry University, Kunming, 650051 Yunnan, China

## Abstract

Electroacupuncture (EA) is a popular therapeutic therapy for premature ovarian insufficiency (POI). However, little has been known about the underlying processes of EA therapy. To investigate the benefit of EA and reveal the mechanism, thirty SD female rats were allocated into the control, model, sham, EA, and GnRHa groups at random. Vaginal smears were used to monitor the rats' estrous cycle. Serum liver and renal function (ALT, AST, BUN, and Cr), sex hormone (FSH, E2, and AMH), oxidative stress markers (SOD, GSH, and MDA), and inflammatory cytokine (IL6, IL1*β*, and TNF*α*) levels were measured by enzyme-linked immunosorbent assay (ELISA). Their ovary morphology was observed by hematoxylin-eosin staining. Transmission electron microscope was used to remark the ultrastructure of the granulocytes. Protein and gene expressions of Keap1/Nrf2/HO-1 pathway were detected by western blot and RT-PCR. Compared with the model group, in the EA group, the levels of serum sex hormones recovered to normal levels. Moreover, it reduced oxidative stress in rats, as demonstrated by increased SOD and GSH levels and decreased MDA levels. Meanwhile, Keap1 mRNA and protein expression dropped considerably in the EA group, while the mRNA and protein expressions of Nrf2 and HO-1 increased. We found that preventive EA might rescue rats with CTX-induced ovarian dysfunction. The anti-inflammatory and antioxidative stress properties of EA, which elevated the Keap1/Nrf2/HO-1 signaling pathway, might be the underlying mechanism. Furthermore, as compared to GnRHa, electroacupuncture did not raise the burden of the liver (ALT and AST) or the kidney (BUN and Cr). Electroacupuncture has a meaningful impact and a sufficient level of safety, making it useful for therapeutic setting in POI.

## 1. Introduction

Premature ovarian insufficiency (POI) [1], formerly known as premature ovarian failure (POF) is a clinical disease characterized by ovarian decline before the age of 40. According to the researchers, the growing morbidity was driven by an increase in the number of premenopausal cancer survivors with iatrogenic POI produced by radiation and chemotherapy. Furthermore, investigations indicated that the rate of chemotherapy-induced permanent infertility ranged from 80% to 100% [2]. Cyclophosphamide (CTX), an alkylating drug with the highest risk of ovarian damage, is indeed commonly used in malignancies such as breast cancer [3]. As per studies, CTX is catalyzed and degraded in the body by liver microsomal enzymes, resulting in the generation of phosphoramide mustard and acrolein, which has cytotoxic effects [4]. During the therapeutic process, blood circulation abnormalities and related body stress injuries might cause a large amount of free radicals to be released. It promotes peroxidation and releases a substantial number of reactive oxygen species (ROS) which will damage the mitochondrial membrane and cell membrane of ovarian granulosa cells, induce an inflammatory cascade, release alarm signals (alarmins), and initiate a cellular response [5]. Granulosa cells in the ovary offer an important environment for the formation and development of egg cells [6]. As a result of the generation of ROS and inflammatory substances, CTX alters follicular growth, oocyte maturation, and apoptosis or atresia in the ovary.

The article "Preventive Electroacupuncture Alleviates Oxidative Stress and Inflammation via Keap1/Nrf2/HO-1 Pathway in Rats with Cyclophosphamide-Induced Premature Ovarian Insufficiency" was retracted in 2023. Reasons: unreliable results or conclusions; concerns about the data; concerns about the peer review; concerns about the citations.

POI is being treated with hormone replacement therapy (HRT) [1], GnRHa intervention [7], assisted reproductive technology (ART), ovarian tissue cryopreservation, and transplantation [8]. However, these approaches have drawbacks such as significant side effects, inconsistency in efficacy, and exorbitant costs [9]. Acupuncture and moxibustion are based on the dialectical theory and general idea of traditional Chinese medicine, and they have the advantages of simplicity, cheap cost, and high efficiency. They also play a vital role in regulating and promoting ovarian function. In 2016, a group consensus on the application of transdermal electrical acupoint activation and electroacupuncture (EA) in infertility treatment was published [10]. Electroacupuncture can control the reproductive endocrine system's function, stimulate the formation of follicles, replenish ovarian reserve, and induce ovulation [11]. In a preliminary clinical trial, we reported that acupuncture might dramatically increase patients' ovarian reserve function [12, 13]. Furthermore, in the preexperiment of modeling the simultaneous acupuncture intervention, the number of primordial and primary follicles risen exponentially in the acupuncture group as compared to the model group. However, its method of action is yet unknown. The Keap1/Nrf2/HO-1 pathway is a significant cellular defense mechanism against the cytotoxic effects of oxidative stress [14, 15], and Nrf2 is a transcription factor that helps to modulate antioxidant responses to stress [16, 17]. Meanwhile, HO-1 and its enzymatic byproducts mediate the resolution of inflammatory reactions and are important inflammatory regulators [18]. We attempted to investigate the therapeutic principle and probable mechanism of electroacupuncture in rats with CTX-induced POI in this study. Electroacupuncture is thought to decrease the inflammatory response in the ovary by activating the Keap-1/Nrf2/HO-1 antioxidant stress signaling pathway. As a result, the onset and development of POI in rats are prevented.

The article "Preventive Electroacupuncture Alleviates Oxidative Stress and Inflammation via Keap1/Nrf2/HO-1 Pathway in Rats with Cyclophosphamide-Induced Premature Ovarian Insufficiency" was retracted in 2023. Reasons: unreliable results or conclusions; concerns about the data; concerns about the peer review; concerns about the citations.

## 2. Materials and Methods

### 2.1. Animals and Experimental Design

30 female Sprague-Dawley rats aged 9 weeks and weighing 240 ± 20 g were purchased from Sino-British SIPPR/BK Lab Animal Ltd. (Shanghai, China). SCXK (HU) 2018-0006 is the certificate number for the animal. All of the animals were kept in the Laboratory Animal Center's grading room, which had a 12-hour cycle of darkness and light and a steady temperature of 21-23°C and was pathogen-free. After a week of adaptive feeding, 6 rats were randomly selected to form the control group, while the other 24 received intraperitoneal injections of CTX (50 mg/kg body weight at D10 and 8 mg/kg body weight from D11 to D25) to create a CTX-induced POI model. Six rats were chosen at random to receive subcutaneous injections of GnRHa (calculated by body surface area, 0.1 mg per time at D1 and D5); the rest of the 18 rats were randomly divided into three groups (*n* = 6 per group): a POI model group, a POI plus sham-EA group, and a preventive electroacupuncture group. The acupuncture sites were chosen based on the rats' acupoint pattern: BL23, Shenshu, the bladder meridian of foot-taiyang; DU20, Baihui, governing vessel; KI3, Tai Xi, the kidney meridian of foot-shaoyin; SP6, San Yinjiao, the spleen meridian of foot-taiyin; ST36, Zu Sanli, the stomach meridian of foot-yangming; and CV4, Guanyuan, conception meridian. Huatuo millineedles (0.19 mm × 10.00 mm, Suzhou Medical Equipment Co., Ltd.) were placed perpendicularly or obliquely into the acupuncture sites listed above, with a depth of 3 mm. Then, the Huatuo electroacupuncture device (SDZ-II, Suzhou Medical Supplies Factory Co., Ltd.) was connected to the needles for 15 min, by using continuous wave, 0.1~1 mA intensity, and 1~3 Hz frequency. The rats in the EA group were treated from D10 to D25. The sham-EA group stimulates the nonmeridian points 1 cm next to the acupuncture point.

The article "Preventive Electroacupuncture Alleviates Oxidative Stress and Inflammation via Keap1/Nrf2/HO-1 Pathway in Rats with Cyclophosphamide-Induced Premature Ovarian Insufficiency" was retracted in 2023. Reasons: unreliable results or conclusions; concerns about the data; concerns about the peer review; concerns about the citations.

We collect the materials from the rats within 24 hours of the treatment period ending. The rats were first sedated with 3% pentobarbital sodium (0.1 ml/100 g body weight) and placed on the sample table. Second, abdominal aortic blood was collected after the abdominal skin of the rats was entirely removed to reveal the inside of the abdomen. The tissue was split in half after the ovaries were weighed, with one half being fixed in 4% paraformaldehyde and 4% glutaraldehyde and the other half being snap-frozen and stored at 80°C for further study.

### 2.2. Determination of Estrus Cycle

From D10 to D25, vaginal swabs were taken to track the estrus cycle. After the smears were stained with HE and the acquired epithelial cells were collected by swabbing the rat's vagina, their morphology was examined under a light microscope (0.1 percent, Solaibao Technology Co., Ltd., Beijing, China).

### 2.3. Enzyme-Linked Immunosorbent Assay (ELISA)

Specific ELISA kits (Nanjing Jin Yibai Biological Technology Co., Ltd., Shanghai, China) were used to measure the levels of serum sex hormones (FSH, E2, and AMH), liver and renal function (ALT, AST, BUN, and Cr), oxidative stress markers (SOD, GSH, and MDA), and inflammatory cytokines (IL6, IL1*β*, and TNF*α*) in accordance with the manufacturer's instructions (A001-3, A006-2, A003-1, JEB-12673, JEB-12597, JEB-10719, and JEB-12991). The absorbance was used to quantify the concentration, and the final result was obtained using the standard curve. Three times were run through each experiment.

### 2.4. Histological Processing and Follicle Count

Ovaries that had been fixed in paraffin were divided into 5 mm histological sections for HE staining, and serial sections were mounted on slides. To evaluate the impact of the chemotherapy on ovarian follicles, follicles were categorized and counted after deparaffinization and rehydration. According to Kalich-Philosoph et al. [19], all follicle counts were carried out by two separate researchers who were unaware of the experimental groups. Ovaries were serially cut into five-micron sections, with every fifth part dyed with HE. Only follicles with an oocyte nucleus that could be seen clearly were scored. Primordial follicles are those that contain an intact oocyte and a single layer of flattened squamous follicular cells. A main follicle was characterized as an expanded oocyte covered in a single layer of cuboidal granulosa cells. Preantral follicles were recognized as oocytes with two or more layers of granulosa cells but no discernible gap between granulosa cells. An oocyte with a clear nucleus, an antrum, and a theca layer were present in antral follicles when scoring was done. Only when a degenerating oocyte and pycnotic granulosa cells were seen were atretic follicles counted. Every fifth section was counted to estimate the number of follicles in each stage, and the total was multiplied by a correction factor of 5 to reflect the entire ovary [20]. The information is shown as the number of follicles at each stage of development (*n* = 6 ovaries per group).

The article "Preventive Electroacupuncture Alleviates Oxidative Stress and Inflammation via Keap1/Nrf2/HO-1 Pathway in Rats with Cyclophosphamide-Induced Premature Ovarian Insufficiency" was retracted in 2023. Reasons: unreliable results or conclusions; concerns about the data; concerns about the peer review; concerns about the citations.

### 2.5. Transmission Electron Microscope (TEM) Staining

1 mm^3^ tissue blocks were fixed with fresh TEM fixative (Wuhan Servicebio Technology Co., Ltd., G1102) at 4°C. And then, wash the tissues using 0.1 M PB (pH 7.4). Tissues stay away from light post that has been 0.1 M PB and 1 percent OsO4 (Ted Pella Inc.) fixed for two hours. Dehydrate at room temperature: 30%-50%-70%-80%-95%-100% ethanol, 20 min each, finally two changes of acetone (Sinopharm Chemical Reagent Co., Ltd., 10000418) for 15 min. Place the tissues within the pure EMBed 812 (SPI, 90529-77-4) and pour the pure EMBed 812 into the embedding models. Then, maintain at 37°C. The samples and embedding models were placed in a 65°C oven to polymerize for more than 48 hours. The tissues were fished out onto the 150 mesh cuprum grids using formvar film after the resin blocks were thinned out to 60–80 nm using the ultramicrotome (Leica, UC7). After 2.6 percent lead citrate, which will prevent CO_2_ staining for 8 minutes, saturated alcohol solution with uranium acetate will do the same. The cuprum grids were dried at room temperature for a whole night. The cuprum grids are viewed and photographed using a TEM (HITACHI, HT7800/HT7700).

### 2.6. Real-Time PCR

Nrf2, Keap1, and HO-1 mRNA expression levels were assessed using quantitative real-time reverse transcriptase PCR (RT-qPCR). The TRIZOL reagent (Invitrogen, 1596-026), together with chloroform extraction and ethanol precipitation, was used to extract total RNA. Reverse transcription kit (Fermentas, #K1622) and total RNA diluted to a standard concentration of 500 ng/mL were combined to create an RT reaction solution. The mixture was then gently mixed, and the ABI-7300 PCR apparatus carried out the reverse transcription process to create cDNA. Then, using an ABI Prism 7300 SDS Software and a PCR reaction mix made up of reverse transcriptional production cDNA and a SYBR Green PCR kit (Thermo, #K0223), RT-qPCR was carried out as directed by the manufacturer. Shenggong Biotechnology Co., Ltd., created primers (Shanghai, China). After polymerase chain reaction, the expression levels of connected genes were examined using the relative quantitative approach and relative standard curve, with each sample being detected, on mean, three times.

The article "Preventive Electroacupuncture Alleviates Oxidative Stress and Inflammation via Keap1/Nrf2/HO-1 Pathway in Rats with Cyclophosphamide-Induced Premature Ovarian Insufficiency" was retracted in 2023. Reasons: unreliable results or conclusions; concerns about the data; concerns about the peer review; concerns about the citations.

### 2.7. Western Blot Analysis

Proteins were extracted from ovarian tissues and quantified using BCA protein assay kits (P0012 BB18091, Beyotime Biotechnology, Shanghai, China). Using an electrophoresis device (mini protean 3 cell, BIO-RAD, USA), an identical amount of protein (20 mg/lane) was electrophoresed on an SDS-PAGE gel (S1010, Solarbio). Then, using the Trans-Blot Turbo Transfer System, the chosen target gel band was transferred to NC membranes (HATF00010, Millipore, Darmstadt, Germany) (PS-9, Dalian Jingmai Technology CO., China). 5% skimmed milk (D8340, Solarbio) was used to block the membranes for an hour at room temperature, and then, the primary antibodies anti-Keap1 (1 : 500, Abcam, Ab119403), anti-Nrf2 (1 : 1000, Abcam, Ab92946), and anti-HO-1(1 : 1000, Abcam, Ab68477) were incubated on the membranes overnight at 4°C. Anti-GAPDH (1 : 2000, #5174) was come from Cell Signaling Technology, Beverly, MA, USA. Before being incubated with the appropriate goat anti-rabbit IgG (H+L) secondary antibody (1 : 1000, A0208, Bi Yuntian Technology Co. China) or goat anti-mouse IgG (H+L) secondary antibody (1 : 1000, A0216, Bi Yuntian Technology Co. China), the membranes were washed with Tris-buffered saline and Tween 20 (TBST). Finally, protein bands (WBKLS0100, Millipore, Darmstadt, Germany) were recognized by enhanced chemiluminescence (ECL) advance reagent and quantified by Tanon Imaging System (Tanon-5200).

### 2.8. Statistical Analysis

The SPSS 26.0 program was used to analyze the data. The information was presented as means and standard deviations (SD). Three different experiments were used to compute the means and SD. The Student's *t*-test was used to compare the differences between the two groups. One-way analysis of variance (ANOVA) was used to compare data from various groups. *p* < 0.05 or *p* < 0.01 indicated that a difference was statistically significant.

## 3. Results

### 3.1. EA Is Effective and Safe

#### 3.1.1. EA Increased Body Weight and the Ovarian Index

As indicated in Figure 1(a), before the experiment, there were no appreciable differences in body weight amongst the five groups (*p* > 0.05). The average body weight of the model group has consistently been lower than that of the control group since D15 (^#^*p* < 0.05 and ^##^*p* < 0.01). Additionally, rats in the EA and GnRHa groups had significantly higher average body weights than the model group after a 5-day course of EA or GnRHa medication ^(^^∗∗^*p* < 0.01, EA group vs. model group; ^@@^*p* < 0.01, GnRHa group vs. model group).  Figure 1(b) demonstrates that the ovarian index massively increased in the EA and GnRHa groups compared to the model group ^(^^∗∗^*p* < 0.01), whereas it considerably decreased in the model group compared to the control group ^(##^*p* < 0.01). Moreover, we discovered that the hair in the model group was frizzy and dull, and the limbs were rather cyanosis. In the EA group, on the other hand, the hair was smooth, and the extremities were warm and rosy.

The article "Preventive Electroacupuncture Alleviates Oxidative Stress and Inflammation via Keap1/Nrf2/HO-1 Pathway in Rats with Cyclophosphamide-Induced Premature Ovarian Insufficiency" was retracted in 2023. Reasons: unreliable results or conclusions; concerns about the data; concerns about the peer review; concerns about the citations.

#### 3.1.2. Acupuncture Could Regulate and Restore the Normal Estrous Cycle Changes in CTX-Induced POI Models

Figure 1(c) shows the estrous cycle of normal rats. There are fewer keratinocytes and leukocytes and more nucleated epithelial cells in proestrum. The oestrum contains a considerable number of keratinocytes, as well as a few nucleated epithelial cells and leukocytes. During the metestrum, keratinocytes, nucleated epithelial cells, and leukocytes exist in equal proportions, while in the diestrum, the number of leukocytes is predominant, with a small amount of nucleated epithelial cells and keratinocytes. Having followed modeling, the rats exhibited periodic disorders including protracted or arrested cycles, a significant decline in the amount of exfoliated keratinized epithelial cells, and leukocytosis. The diestrum or metestrum was where the majority of the rats that were successfully modeled were found. Following therapy, the estrous cycles of the EA group and GnRHa group gradually returned to normal in comparison to the model group (Figure 1(d)).

#### 3.1.3. Preventive Electroacupuncture Repaired the Concentration of Serum Sex Hormones

Serum AMH and E2 levels in the model group were lower than those in the control group, whereas FSH levels were higher ^(##^*p* < 0.01). In the EA and GnRHa groups, the levels of AMH and E2 rose after treatment with medications or electroacupuncture, whereas the level of FSH reduced (^∗∗^*p* < 0.01) (Figures 1(e)–1(g)).

#### 3.1.4. Preventive Electroacupuncture Did Not Aggravate the Kidney-Liver Burden

Cyclophosphamide was clearly harmful to the liver and kidney, the serum ALT, AST, and Cr were markedly elevated (^##^*p* < 0.01). In comparison to GnRHa, the EA group did not raise the strain on the liver and kidney (^@@^*p* < 0.01) (Figure 2).

### 3.2. EA Treatment Improves Ovarian Morphology and the Ultrastructure

#### 3.2.1. EA Played a Crucial Role in the Development and Ovulation of Follicles at All Levels

Figure 3 shows that the model rats' ovarian morphology was atrophied to some extent (*p* > 0.05), the ovarian cortex thickened, and the structure was disordered as compared to the control group. The number of ovarian primordial follicles, primary follicles, secondary follicles, mature follicles, and corpus luteum dropped considerably (^#^*p* < 0.05 and ^##^*p* < 0.01), but atresic follicles and interstitial fibrosis increased. Fundamentally, ovarian morphology restored during EA or GnRHa treatment, ovarian follicle phases and corpus luteum rose (^∗^*p* < 0.05 and ^∗∗^*p* < 0.01), and the number of atresic follicles significantly decreased (^∗∗^*p* < 0.01).

The article "Preventive Electroacupuncture Alleviates Oxidative Stress and Inflammation via Keap1/Nrf2/HO-1 Pathway in Rats with Cyclophosphamide-Induced Premature Ovarian Insufficiency" was retracted in 2023. Reasons: unreliable results or conclusions; concerns about the data; concerns about the peer review; concerns about the citations.

#### 3.2.2. EA Treatment Preserved the Normal Ultrastructure of Ovarian Granulosa Cells

There were variations in ovarian granulosa cells between the groups. Granulosa cells in control group (Figure 4(a)) had regular nuclei, uniform chromatin, plenty of mitochondria, and endoplasmic reticulum. A sizable portion of the granulosa cells in the ovary of the model group (Figure 4(b)) had experienced severe damage, including altered nuclear morphology, aberrant chromatin condensation, mitochondrial vacuoles, and cell matrix edema. When compared to the model group, the EA and GnRHa groups (Figures 4(d) and 4(e)) displayed symmetrical nuclei, evenly arranged chromatin, and more and fully constructed mitochondria.

### 3.3. Electroacupuncture Reduced Oxidative Stress and Inflammation in POI Rats Caused by Cyclophosphamide

Oxidative damage occurred in the model group, and the release of inflammatory factors increased. In contrast, the oxidative stress marker MDA was severely decreased in the serum of rats in the electroacupuncture group (Figure 5(a)), while the antioxidant stress indicators SOD and GSH were enhanced (Figures 5(b) and 5(c)). Simultaneously, in the oxidative stress signaling pathway, Keap1 mRNA and protein contents dropped, while Nrf2 and HO-1 mRNA and protein contents considerably increased (Figures 5(d)–5(f)). Finally, blood levels of the HO-1-associated inflammatory factors IL6, IL1*β*, and TNF*α* declined (Figures 5(g)–5(i)).

## 4. Discussion

The ovaries are extremely sensitive to the chemotherapy medications. Female tumor patients would have substantial ovarian function impairment after using chemotherapy medicines, resulting in a loss in ovarian reserve, which in turn leads chemotherapy-induced premature ovarian failure. Cyclophosphamide is a multifunctional alkylating agent that is commonly used in the treatment of breast cancer, ovarian cancer, lung cancer, multiple myeloma, and other tumor conditions. Simultaneously, its reproductive toxicity has garnered increasing attention. Excess germinal primordial follicles, inadequate development of follicles at all stages, and follicular pool depletion result in diminished ovarian reserve [3]. Previous studies have shown that its mechanism is mainly through oxidative stress damage, affecting hormone levels, and inducing germ cell apoptosis [5]. Based on the literature, we established a CTX-induced chemogenic POI rat model [21] and investigated the effect of preventative acupuncture on the Keap/Nrf2/HO-1 pathway in the pathogenic phase of POI. Concurrently, we picked GnRHa [7], a regularly used medicine for POI, which mechanism is similar to that of electroacupuncture in that it inhibits the production of follicle-stimulating hormone, inhibits the growth of follicles, leaves them in a dormant condition, and prevents the attack of chemotherapy medications, as the positive drug control group and nonmeridian points as the sham electroacupuncture group. Our findings demonstrated that CTX caused the emergence and progression of POI, including substantial reductions in body weight and ovarian index, disruption of the estrous cycle, irregular levels of sex hormones, and altered ovarian morphology, all of which were consistent with earlier research [21, 22]. Preventive electroacupuncture and GnRHa could both considerably relieve the symptoms listed above while decreasing oxidative stress and inflammatory reactions. It is worthy of note that electroacupuncture had no negative effects on the liver or renal functions in POI rats.

The article "Preventive Electroacupuncture Alleviates Oxidative Stress and Inflammation via Keap1/Nrf2/HO-1 Pathway in Rats with Cyclophosphamide-Induced Premature Ovarian Insufficiency" was retracted in 2023. Reasons: unreliable results or conclusions; concerns about the data; concerns about the peer review; concerns about the citations.

First of all, we discovered that EA therapy boosted the body weight and ovarian index of CTX-induced POI rats. Further to that, by histomorphology and ultramicrostructure, we discovered that the number of primordial follicles, primary follicles, secondary follicles, antral follicles, and corpus luteum increased significantly, while the number of atretic follicles decreased. Granulosa cells were well aligned with intact membranes, relatively normal mitochondrial morphology, and reduced damage. These findings indicate that EA dramatically increased folliculogenesis, ovulation, and follicle quality in POI rats. AMH is released by the granulosa cells of developing follicles and is recognized as a valid biological measure of ovarian reserve [23]. CTX was shown to lower the serum AMH concentration in our study. EA therapy, in essence, reversed this impact, implying that EA might protect ovarian reserve function by improving ovarian granulosa cells. The estrous cycle, which is governed by the hypothalamus-pituitary-ovarian axis, changes monthly due to sex hormone fluctuations. FSH is a gonadotropin emitted by the antehypophysis that drives follicle growth, development, and maturation [24, 25]. Due to the obvious reduction in ovarian reserve and follicle count, estrogen and progesterone are ineffective to restrict pituitary FSH secretion, resulting in higher blood FSH levels. E2, which is generated by FSH-stimulated granulosa cells, enhances follicle growth and development while developing a low feedback impact on the hypothalamus and pituitary glands. When a patient's serum E2 level is lower, it causes aberrant follicular formation, reduces ovarian function, inhibits negative feedback, and inappropriately raises FSH levels. The estrous cycle was delayed or disrupted as a result of the modeling, the FSH level risen exponentially, and the E2 level reduced greatly. Both of these results revealed that CTX is toxic to the gonad of rats and impairs the hypothalamus-pituitary-ovarian axis, resulting in insufficient hormone levels expressed to sustain the periodic alterations of vaginal exfoliated cells. The concentrations of FSH and E2 were restored in the EA group, and the estrous cycles were mostly normal, illustrating that acupuncture might modify neuroendocrine function and balance hormone secretion.

The article "Preventive Electroacupuncture Alleviates Oxidative Stress and Inflammation via Keap1/Nrf2/HO-1 Pathway in Rats with Cyclophosphamide-Induced Premature Ovarian Insufficiency" was retracted in 2023. Reasons: unreliable results or conclusions; concerns about the data; concerns about the peer review; concerns about the citations.

Oxidative stress has been linked to the loss in ovarian reserve produced by chemotherapy treatments, according to research [26, 27]. MDA, SOD, and GSH, which are oxidative index-related enzymes, are routinely employed markers to assess the degree of oxidative damage. MDA is a byproduct of oxidative stress. MDA, as a byproduct of lipid peroxidation, can indicate the degree of oxidative damage, and it is cross-linked with biological macromolecules such as nucleic acids and proteins to denature and inactivate them. SOD is an essential antioxidant defense enzyme that initiates a disproportionation process that transforms superoxide anion to hydrogen peroxide. By catalyzing reduced glutathione, GSH resists the reduction process of hydrogen peroxide, eliminates lipid peroxides and hydrogen peroxide, and decreases the body's oxidative damage [28]. The ovary's oxidative stress response is also aided by proteins in the Keap-1/Nrf2/HO-1 signaling pathway. Nrf2 is a critical component in initiating endogenous defense against oxidative damage. While activated by oxidative damage, Nrf2 and its cytoplasmic binding proteins, in collaboration with Kelch-like epichlorohydrin-associated protein-1 (Keap1), bind to antioxidant response elements (AREs) in target gene promoters, promoting transcription of the antioxidant gene HO-1 and thus protecting cells [14, 15, 29]. It has been proven experimentally that Nrf2 is an essential sensor and regulator of chemical homeostasis in ovarian cells and that it can protect ovarian cells against aggressiveness by managing metabolic detoxification and exerting an endogenous antioxidant effect [16, 30, 31]. The findings of this investigation revealed that the activities of SOD- and GSH-related ovarian oxidation markers in the model group declined, while the amount of MDA increased, indicating that the ovarian tissue of POI model rats sustained oxidative damage. The expression of Keap-1 protein in ovarian tissue rose, whereas Nrf2/HO-1 protein expression decreased, which is consistent with previous results. It is speculated that CTX may cause oxidative damage in the ovary. In addition, the inflammatory response leads to ovarian follicular loss [32]. An increasing amount of evidence shows that excessive inflammation may disrupt normal ovarian follicular dynamics, hence leading to infertility [33, 34]. The levels of IL6, IL1*β*, and TNF*α* in serum increased, indicating that the POI rats had inflammatory infiltration. After electroacupuncture treatment, SOD and GSH increased, MDA decreased, Keap1/Nrf2/HO-1 endogenous antioxidant stress response was enhanced, and inflammatory response was reduced in rats (Figure 6).

The article "Preventive Electroacupuncture Alleviates Oxidative Stress and Inflammation via Keap1/Nrf2/HO-1 Pathway in Rats with Cyclophosphamide-Induced Premature Ovarian Insufficiency" was retracted in 2023. Reasons: unreliable results or conclusions; concerns about the data; concerns about the peer review; concerns about the citations.

POI falls under the categories of “infertility” and “amenorrhea” in TCM. The kidney, spleen, and liver are all involved in reproduction. The kidney stores life's essence and regulates growth, development, and reproduction. The spleen and stomach serve as a source of qi and blood production and transformation. Blood is stored in the liver. When qi and blood appear to be inadequate, and the Chong and Ren meridians are harmed, infertility occurs. As a consequence, TCM treatment focuses mostly on the liver, spleen, and kidney. In this study, we use Shenshu (BL23) with Taixi (KI3) to invigorate the kidney qi, replenish the kidney yin, strengthen the kidney yang, and nourish the uterine collaterals [35]. Both Guanyuan (CV4) and Sanyinjiao (SP6) have close connections with the three yin meridians of foot and the two meridians of Ren and Chong. They are the key points to boost the production of qi and blood and nourish the uterine collaterals by regulating the liver, spleen, and kidney. A vast number of studies suggested that these two may stimulate estrogen secretion, block hypothalamic and pituitary control of gonadotropins and gonadotropin-releasing hormone, and had a beneficial influence on the HPO axis [36, 37]. Finally, we added Baihui (DU20) to smooth the liver and tranquilizing the mind, and motivated Zusanli (ST36) to tonify the foundation of postnatal life [38]. Furthermore, we advance the treatment node and provide acupuncture intervention concurrently with chemotherapy, in accordance with the theory of “preventive treatment” of traditional Chinese medicine, in order to counteract the cumulative effect of the toxicity of CTX and its metabolites, effectively protect the ovarian reserve function as soon as possible, and prevent the occurrence and development of POI. Moreover, our study, which was based on traditional acupuncture, used neurophysiology principles to regulate nerve endings and immunological variables by adequate electrical stimulation, which might boost ovarian perfusion, regulate sympathetic nerve activity, and influence endocrine [39, 40]. Electroacupuncture therapy blends conventional acupuncture therapy with electrophysiological theory in order to measure and standardize stimulation and increase disease effectiveness. The most essential point is that acupuncture has gained worldwide acceptance. Acupuncture offers unsurpassed safety benefits over western medication and traditional Chinese herbs because it bypasses liver and renal processing and directly activates organelles or cytokines to accomplish therapeutic effects [41, 42]. Simultaneously, acupuncture and moxibustion focus on overall regulation and multitarget treatment. It provides significant benefits in a variety of conditions, including infertility, neurological diseases, and immune system disorders. Our study provides scientific evidence for the beneficial effects of EA, paving the way for possible clinical trials in the future.

The article "Preventive Electroacupuncture Alleviates Oxidative Stress and Inflammation via Keap1/Nrf2/HO-1 Pathway in Rats with Cyclophosphamide-Induced Premature Ovarian Insufficiency" was retracted in 2023. Reasons: unreliable results or conclusions; concerns about the data; concerns about the peer review; concerns about the citations.

## 5. Conclusion

In summary, this study looked at the effectiveness and mechanism of electroacupuncture in the treatment of CTX-induced POI in rats. Preventive electroacupuncture controls hormone levels via the hypothalamus-pituitary-ovarian axis, regulates the estrous cycle in rats, decreases inflammation, improves oxidative stress, and improves ovarian function. Our research offers a fresh viewpoint and a solid foundation for the therapeutic treatment of POI.

## Figures and Tables

**Figure 1:** (a) Rats weight (g). (b) Ovarian index (mg/g). (c and d) The estrous cycle of rats during D10 to D25: vaginal smears were examined by HE staining in each group (×200 magnification; scale bars: 10 *μ*m). (e–g) EA upregulate serum AMH and E2 levels and downregulate serum FSH Levels in POI rats. (e) Serum AMH, (f) serum FSH, and (G) serum E2. Values were presented as mean ± SD (*n* = 6; ^#^*p* < 0.05 and ^##^*p* < 0.01, compared with the control group; ^∗^*p* < 0.05 and ^∗∗^*p* < 0.01, the EA group versus the model group; ^@^*p* < 0.05 and ^@@^*p* < 0.01, the GnRHa group versus the model group). HE: hematoxylin and eosin; SD: standard deviation.

**Figure 2:** Effects of EA on liver enzymes (ALT and AST) and kidney functions (BUN and Cr). Modeling was harmful to the liver and kidney. Compared to GnRHa group, the EA group did not raise the strain on the liver and kidney (^##^*p* < 0.01, compared with the control group; ^∗^*p* < 0.05 and ^∗∗^*p* < 0.01, compared with the model group; ^@@^compared with the EA group).

**Figure 3:** Hematoxylin and eosin (H&E) staining of ovarian tissues. (a) Follicle cells: A: primordial follicle, B: primary follicle, C: secondary follicle, D: mature follicle, E: atresic follicle, F: corpus luteum. (b) Ovarian tissues: A: control group, B: model group, C: sham group, D: EA group, and E: GnRHa group. (c) Follicle count. The values were shown as mean ± SD (*n* = 6; ^#^*p* < 0.05 and ^##^*p* < 0.01, in contrast to the control group; ^∗^*p* < 0.05 and ^∗∗^*p* < 0.01, in contrast to the model group).

The article "Preventive Electroacupuncture Alleviates Oxidative Stress and Inflammation via Keap1/Nrf2/HO-1 Pathway in Rats with Cyclophosphamide-Induced Premature Ovarian Insufficiency" was retracted in 2023. Reasons: unreliable results or conclusions; concerns about the data; concerns about the peer review; concerns about the citations.

**Figure 4:** The ultrastructure of ovarian granulosa cells was observed under transmission electron microscope (×2000/5000 magnification). (a) Control group, (b) model group, (c) sham group, (d) EA group, and (e) GnRHa group. N: nucleus; M: mitochondria.

**Figure 5:** (a) The level of oxidative stress marker MDA. (b and c) The level of antioxidant stress indicator SOD and GSH. (d and e) The expression of the Keap1/Nrf2/HO-1 pathway maker proteins in ovarian tissues was observed using western blot. (d) The representative immunoblots. (e) The expression was quantitated using ImageJ software. (f) Effect of electroacupuncture on the expression of the gene in Keap1/Nrf2/HO-1 signaling pathway in ovarian tissues. (g–i) The level of proinflammatory factor: (g) IL6, (h) IL1*β*, and (i) TNF*α*. Values are presented as means ± SD (^#^*p* < 0.05 and ^##^*p* < 0.01, in comparison to the control group; ^∗^*p* < 0.05 and ^∗∗^*p* < 0.01, in comparison to the model group).

**Figure 6:** Schematic diagram of EA regulating antioxidant stress and inflammatory response in POI rats (by Figdraw: http://www.figdraw.com/).

## Data Availability

The data used to support the findings of this study are available from the corresponding author upon request.
